# Energy-Efficient Cluster Formation in IoT-Enabled Wireless Body Area Network

**DOI:** 10.1155/2022/2558590

**Published:** 2022-04-05

**Authors:** Asim Zeb, Sonia Wakeel, Taj Rahman, Inayat Khan, M. Irfan Uddin, Badam Niazi

**Affiliations:** ^1^Department of Computer Science, Abbottabad University of Science and Technology, Abbottabad 22010, Pakistan; ^2^Department of Physical and Numerical Science, Qurtuba University of Science and Information Technology, Peshawar 2500, Pakistan; ^3^Department of Computer Science, University of Buner, Buner 19290, Pakistan; ^4^Institute of Computing, Kohat University of Science and Technology, Kohat 26000, Pakistan; ^5^Department of Computer Science, University of Nangarhar, Nangarhar 2600, Afghanistan

## Abstract

Wireless sensor network is widely used in different IoT-enabled applications such as health care, underwater sensor networks, body area networks, and various offices. A sensor node may face operational difficulties due to low computing capacity. Moreover, mobility has become an open challenge in the healthcare wireless body area network that is highly affected by message loss due to topological manipulation. In this article, an enhanced version of the well-known algorithm MT-MAC is proposed, namely DT-MAC, to ensure successful message delivery. It considers node handover mechanism among virtual clusters to ensure network integrity and also uses the concept of minimum connected dominating set for network formation to achieve efficient energy utilization. It is then compared with well-known algorithms such as MT-MAC. The simulation results show that an increase in little latency of roughly 3 percent in using the proposed protocol improves the MT-MAC's packet delivery by 13–17 percent and the response time by around 15 percent. Therefore, the algorithm is best fitted for real-time applications where the high packet delivery and response time are required.

## 1. Introduction

A wireless body area network (WBAN) is an example of human and machine connectivity. As per the IEEE 802.15.6 : 20121 standards, a WBAN is “a connectivity standard designed for low-power devices to cover a range of uses, including medical, consumer electronics or personal entertainment and other applications, for their function on, in or around the human body (but not limited to humans).” Via the use of IoT-based sensor nodes, WBANs are able to track physiological vital signals at any moment, anywhere through the Internet. Small sensor sizes are comfortable to use and do not conflict with normal activities in life [1–4]. The doctor or hospital is notified early until the real event takes place by a properly defined BAN. If any unusual adjustments are detected, various types of warnings or alerts are being used to notify the doctor. In time, medication can save a precious life and increase the quality of life for public. These heterogeneous IoT-based WBANs have a huge opportunity for future healthcare implementations to deliver an enormous revolution [5–9]. These networks are expected to bring about a significant improvement in disease prevention and control procedures for increased procurement. For the cause of mankind, WBAN is a marvelous use of information technology [10–12]. Sensed data from multiple heterogeneous sensor nodes are communicated towards a central point (sink) in case of any abnormality and are eventually be transmitted over the Internet to an emergency care centre. Doctors would be able to make better choices when they collect evidence from the end user's natural living environment. This remote patient control would allow them the ability to resume their regular operations rather than remaining at home or in a hospital [13–15]. IoT-based sensor networks are not without difficulties, and higher throughput, minimal latency, longer network life, and lower energy usage for improved performance are typical challenges [12, 14, 16–18]. Sensor nodes are mostly fitted with minimal battery supply due to size limitations and portability problems. In these networks, network lifespan plays a vital role as systems are required to operate over a longer period of time [19]. WBANs have restricted channel capacity and buffer space, apart from the limited availability of batteries. Sensors would also have two types of priority-level data packets, one being the usual data detected and the other being emergency or life-critical data [20–22]. High priority, less delay, and error-free data transmission under specified time limits [23, 24] are needed for life-critical data. The working theory of sensor networks is focused on event-driven strategy and refers to many-to-one interaction [25–27]. The nodes closest to the sink have a higher rate of packet arrival than their service rate, which creates congestion at the node level (buffer overflow). Network life and capacity would also be diminished. Clustering, which is a hierarchical representation of the network, is one of the most successful strategies to address those difficulties. In clustering, each cluster consists of the head of the cluster and each cluster node is grouped into a fitting cluster [28, 29]. An important role of cluster head is to provide a communication between sensor nodes and the base station efficiently [30]. Diverse techniques are recently proposed to overcome the challenges of limited energy, namely S-MAC, T-MAC, MS-MAC, and MT-MAC [31–34].

There are three types of nodes in MT-MAC algorithm, namely cluster member, cluster head, and border node [35]. The border node listens to both clusters and eventually dissipates energy consumption rapidly. However, there is no consideration of minimizing the border nodes to achieve a longer lifetime. We use the idea of a minimum connected dominating set (MCDS) among all connected dominating sets to minimize the border nodes. Maintaining the minimum cardinality among all MCDS requires careful consideration to improve the current MAC techniques [16]. Moreover, among entire, idle hearing is the best important basis of energy dissipation. Idle listening waists energy drastically when a responder node keeps its radio on to listen to the channel for expected data frames, while there is no sender node. Both the mentioned scenarios, such as minimizing border nodes and idle listening, are taken into consideration in DT-MAC. Since the radio is controlled by MAC, governing the power consumption through improvement in MAC protocol can significantly increase the lifetime of the power sources in a WSN.

Wireless technology is moving towards healthcare and emergency-related applications such as structural health monitoring and assisting elderly citizens health, and mobility has become a new era that needs further exploration in WSNs. Currently, MAC protocols nearly abandon the importance of such considerations, yet an efficient MAC protocol requires implementable schemes under mobility.

Timeout MAC (T-MAC) deploys dynamic active time in flexible load that decreases the idle period. The algorithm also regulates every node sleeping manner as no activation in defined time. According to alteration in data load, T-MAC employs an adaptive and dynamic schedule. Similarly, S-MAC and T-MAC split the network into many virtual clusters to minimize the control overheads. Such clustering techniques lead to efficient use of the network resource in terms of energy depletion, least delay, and efficient bandwidth utilization [32, 33]. MT-MAC is one of the well-known energy-efficient MAC protocols that have resulted that MT-MAC achieves well under stationary and mobile nodes in the network and it gives efficient results than T-MAC and S-MAC. However, the performance of the algorithm is highly degraded in maintaining MCDS and updating schedules. In MT-MAC, the border node (BN) adopts both virtual schedules and listens to both virtual clusters. Every mobile node can act as border node as soon it listens to both clusters. Therefore, there are more border nodes and it also requires wakeup two times to listen to both clusters. This leads to faster depletion of energy as compared to other nodes in the network. Despite the fact that the performance of MT-MACs has been evaluated in several scenarios, however, the effectiveness of MT-MAC in preserving MCDS in a dynamic context has yet to be evaluated in this article. Thus, a dynamic environment is considered for this study to evaluate the performance of MT-MAC in mobile and permanent nodes coexist. Furthermore, MCDS is considered to achieve an energy-efficient method and dynamic up-gradation of scheduling in MT-MAC protocol, which is known as DT-MAC. The idea behind achieving MCDS considers that a node (*x*) has a schedule and receives a synchronization packet from another node that is different from the current. Now, the node *x* informs its cluster head about that SYNC message from other virtual clusters. The cluster head checks that either the respective virtual cluster is connected through BN or not. When the neighboring virtual cluster is connected through border node, the *x* becomes the cluster member of one of the CH and sets node type to ST. Otherwise, the *x* node sets its node type BN. The BN adopts both schedules and listens to both VCs in its neighborhood. After getting the primary scheduling process, nodes in every single virtual cluster are distributed into three different categories, namely gateway node (GN), cluster head (CH), and stationary node (SN).

Afterwards, the paper's structure is as follows: Section 2 presents an inclusive argument on four popular MAC protocols, namely S-MAC, T-MAC, MS-MAC, and MT-MAC protocols. An enhanced mobility-aware MAC scheme, based on the MT-MAC protocol, is suggested in Section 3. In Section 4, the simulation-based performance assessment results and their discussion were presented, and finally, Section 5 presents an inclusive argument on the presented technique and a conclusion of this article is described.

## 2. Literature Review

There are two types of wireless sensor networks, namely flat network and cluster-based network.

### 2.1. Flat and Cluster-Based Wireless Sensor Network

In a flat network, node functionality and status are the same, where each node acts as a router and also a data generator. However, the network is inefficient in energy-saving, when the size of the network is increasing and also performance.

The large wireless sensor network is divided into small groups such as cluster-based network which generates scalable resutls. There are numeruous advantages of cluster-based wirless sensor network over the flat networks as cluster-based networks reducing communication overhead, minimizing delay and energy depletion which resultantly extends the network lifetime [36–38].

### 2.2. Mobility-Aware Sensor MAC (MS-MAC)

MS-MAC is used to handle mobility based on the actual mobility position of nodes. Every node received signal level messages periodically and in synchronized way from its neighbors' nodes [33].

### 2.3. Timeout MAC (T-MAC)

Timeout MAC (T-MAC) is suggested by Van Dam and Langendoen that deploy dynamic active time in flexible load that decreases the idle period. The algorithm also regulates every node sleeping manner as no activation in defined time. According to alteration in data load, T-MAC employs an adaptive and dynamic schedule. Similarly, S-MAC and T-MAC split the network into many virtual clusters to minimize the control overheads [32].

### 2.4. Energy Conservation in WSN by Differentiating Data Delivery

Packets are dropped in the wireless sensor network when congestion happens. Energy depletion in these transmissions decreases the wireless sensor network lifetime [39]. In a wireless sensor network, successful event detection required timeliness and reliability, and the data delivery is not the same in congestion in a wireless sensor network. Congestion-aware routing exposes the network congested zone, which exists between data sink and high priority data source, and simple forwarding rules are used in the network. Similarly, congestion-aware routing also calculates high priority traffic share rate in congestion for improving enery conservancy in wirelss sensor network [40].

### 2.5. Energy-Efficient Clustering Scheme in WSN

The energy-efficient clustering scheme (EECS) for wireless sensor networks is addressed, which is well suitable for data gathering in the network. The algorithms select CHs with more remaining energy through local radio communication, whereas achieving better CH distributes the network [38, 41].

### 2.6. Mobility-Aware Timeout Medium Access Control Protocol (MT-MAC)

The improved version of T-MAC protocol also called MT-MAC protocol is presented in [34]. Changing the LQI and RSSI values of the received synchronization packets and investigating the mobility of packets, a moveable node is smoothly transferred to another virtual cluster VC without connection losing with other nodes. In T-MAC, MS-MAC solves a high packet delivery ratio, however the MT-MAC outperformed.

Thus, in MT-MAC, the border node (BN) adopts both virtual schedules and listens to both virtual clusters in the immediate vicinity. Every mobile node can take hold as border node. There are more border nodes, and it requires wakeup two times. Consequently, the BN may deplete the energy quicker as compared to other nodes in the network. Thus, the overall network lifetime may suffer a lot due to faster BN energy depletion. The number of BN minimization may eventually increase the network lifetime. Since the BN listens to both clusters and walkups more than one time, decreasing border node eventually increases the lifetime of the network.

## 3. Methodology

### 3.1. Network Model

The following are the considerations for DT-MAC.

Each node is fitted with only one transceiver, such that sending and receiving operations cannot be done concurrently by the node. The communication range of each node is identical if the communication range is assumed to be the maximal distance between the two nodes, such that the transmitted data can be received accurately by the two nodes.

Moreover, in the network, node(s) that is within the communication range of other node(s) is(are) represented by neighbor nodes. In the proposed network model, every node is fitted with a timer which shows the overall waiting period for acceptance of packets. The timer gives time reference to a node to start transmission. When the node modifies the existing cluster, it synchronizes the timer with the new cluster.

Q represents the parent node of the static node in the proposed DT-MAC algorithm. The travelling node (MN) represents a node whose RSSI and LQI values fluctuate between the received SYNC packets. The state of a static node is defined in the cluster member (CM), cluster head (CH), and boundary node (BN). Either CH or GW is the parent node, whereas either CM or CH is the child node. The network's configuration is defined below.

Let *G* = (V, E) be the undirected graph describing a network of wireless sensors, whereby V is the group of nodes reflecting the nodes of the sensor and *E* is the edge set. *u* and v nodes have an edge between them during *G* if they are in the propagation range of each other and only if there is no fluctuation in RSSI and LQI values. *G* nodes in the cluster-based architecture are divided into groups representing clusters. There is one head node in each cluster, called the cluster head (CH), which is linked to all other nodes in its group, called the cluster member (CN). A cluster head and a part of the cluster form a star topology within each group. In graph *G*, no two cluster heads are neighbors and are connected by a single node called the boundary node (BN). As defined in Figure 1(a), a BN links two or more adjacent cluster heads or other BNs. Figure 1(a) defines the shape of the DT-MAC flat network architecture (*G*) (Figure 1(a)). A DT-MAC backbone, denoted as BT(*G*), is a DT-MAC subtree generated by CHs and GWs [19]. A minimal connected dominating set (MCDS) of a BT(*G*) graph is a connected dominating set among all connected dominating sets of BT(*G*) with the smallest possible cardinality (*G*).

The number of vertices in the minimum connected dominant set is the related dominance number of BT(*G*). Since the BT node listens to all VCs, the energy depletes more rapidly than other nodes. Therefore, minimizing the BN via using the concept of MCDS, ultimately longer the lifetime of the network is described in the next section.

### 3.2. Network Model

The following are the considerations for DT-MAC.

Each node is fitted only with single transceiver, such that sending and receiving operations cannot be done concurrently by the node. The communication range of each node is identical if the communication range is assumed to be the maximal distance between the two nodes, such that the transmitted data can be received accurately by the two nodes. In addition, in the network, the node(s) represented by adjacent nodes are within the contact range of other node(s). Each node in the proposed network model is fitted with a timer which shows the overall waiting period for acceptance of packets. The timer gives time reference to a node to start transmission. Once the node changes the current cluster, its timer is synchronized with the new cluster.

The proposed algorithm is based on the scheduling process, which utilizes the “make before split” principle to move mobile nodes to another virtual cluster from one virtual cluster. Similar to MT-MAC, the proposed device initiates the scheduling process, and SYNC with neighbors is maintained by nodes waking up at random times and listening to the media. Similar to the MT-MAC algorithm, a mobile node that leaves its virtual cluster VC and enters into another VC is either cluster member (CM), border node (BN), or cluster head node (CH). These nodes can be stationary if it does not change their position compared with other nodes. Initially, after a specific length of time, the nodes awoke. No SYNC packets are received from the neighboring nodes of node (*x*). It selects a time window and broadcasts a SYNC packet. Moreover, the nodes declare itself as a cluster head node (CH) to neighbor nodes and set its node type to the stationary node. However, *x* has no SYNC packet and receives a SYNC packet from CH and responds a handover bit (HB) to the respective CH. When the CH receives the HB, it sets a time slot for the neighbor node and sends the SYNC packet. Thus, the node becomes the cluster member (CM) of that particular CH and sets node type to the stationary node (ST). Conversely, x.status = MN shows the status of the mobile node and also receives a SYNC packet with a different schedule from another CH (Algorithm 1).

Now, *x* sends a message inquiry to its parent node x.parent about the SYNC packet. The parent checks whether it is connected to other virtual clusters through BN or not.

When it is connected through a border node with other VC, *x* does not change its status, which eventually decreases the number of BN, unlike MT-MAC. Otherwise, *x* sets its node type to BN and adopts both schedules. It means that this specific node wakes up and listens to the two VCs in its immediate area. After getting the initial scheduling process, nodes in each VC are divided into three different types, namely cluster head (CH), border node (BN), and stationary node (SN). The scheduling process is described in Algorithm 1, after considering the following definition. Then, the protocol commences the mobility phase that is shown in Algorithm 2. When the node detects any changes in the RSSI and LQI values of the received SYNC packet, the node flag is changed to the mobile node (MN) and the node activates a timer, such as MT-MAC, when the stationary node (SN) listens to the medium.

If the node persists in the same cluster, after *T* enters the period, the NT flag value of the MN flag is restored to its previous value. Depending on the programme, the amount of the timer is predefined. Unlike MT-MAC, after *T* units of time, the mobile node (*y*) may reach to border node (BN), and the BN sends a message, namely MobileInfo to y.parent and the neighbor nodes. Upon receiving the message to y.parent (cluster head) and potential parent node (*z*), then two operations are performed, one is in y.parent and the other-one is in *z* node. Since the time slot for y.parent is empty, the time slot is deleted upon receiving the message. Secondly, the *z* node reserves a time slot for *y* node upon the message. Next, the nodes *y* and *z* send SYNC message to let the neighbor node know about the updated time slots. When the SYNC message is received to their associated cluster members, their scheduling is updated, respectively. Thus, the neighbor VC can also obtain a replica of the neighbor VC schedule and adopts its schedule and the schedule of the neighbor VC as well. In this case, the MN works much like a wanderer BN, which avails it to have a smooth handover to another VC. The nodes reset the timer that is depending upon the application.

## 4. Results and Discussion

### 4.1. Performance Evaluation

MS-MAC protocol proposes the mobile node that tracks VC border, the node, and its neighbor nodes from an active zone [42]. Equation (1) can be evaluated by the handover ratio.

(1) $$\begin{array}{c} \frac{1}{\mu }=\frac{X}{2v}=>\mu =\frac{2v}{X}. \end{array}$$

*μ* represents the ratio of transferring, *X* represents the VC length, the average velocity of the nodes is represented by V. Consider the case of a network with 49 nodes that have been designed that are equally distributed in 150 × 150 m2 where the location of the network is separated into 4 equivalent VCs. The overall mobile nodes in the network are 20 percent per 5 m/s, and the normal speed is 20 m. (2) can be evaluated by the handover ratio.

(2) $$\begin{array}{c} \mu =2\times \frac{5}{75}=>\mu ≃0.13. \end{array}$$

The network handover is evaluated in the base of (2), where 20 percent of 49 nodes are moveable:

(3) $$\begin{array}{c} \mu \times \frac{20}{100}\times 49≃1.3,\frac{\text{Transfer}}{\text{s}}. \end{array}$$

The assuming network, 1.3 transfer, happens during every single (*s*).

According to [43, 44], equations (4) and (5) are used for evaluating one-hop and two-hop network density, respectively.

(4) $$\begin{array}{c} \rho =\frac{N\pi r^{2}}{A}, \end{array}$$

(5) $$\begin{array}{c} \rho =\frac{N\pi 4r^{2}}{A}, \end{array}$$

where N is the total number of nodes in the network, *r* is the broadcast range of every single node, and A represents the size of the zone where the network is developed.

(6) $$\begin{array}{c} \rho =49\times \pi \times 20^{2}÷150\times 150=>\rho ≃3\left(1-\text{ hop density}\right), \end{array}$$

(7) $$\begin{array}{c} \rho =49\times \pi \times 4\times 20^{2}÷150\times 150=>\rho ≃11\left(2-\text{hop density}\right)\text{.} \end{array}$$

(3) Every single transfer happens in the network; (7) MT-MAC contains an enormous number of nodes in the transfer procedure. Nodes perform synchronization frequently inside the active zone (depending on the speed); as a result, it leads to conserve more energy depletion. Indifference, one-hop neighbors use MT-MAC (6) and it does not contain nodes in the energy depletion procedure. It transfers the mobile node to another VC through a transformation of the flag to every node (for helping the GN distinguish moveable nodes) and notifies the moveable node about the new VC schedule. This method is used in helping with maintenance for the network connectivity, except using the large amounts of memory resources and energy [45–47].

### 4.2. Performance Metrics and Simulation Model

According to the wireless sensor network (WSN) with a mobile node, the performance of a simulator can be conducted with the proposed enhancement schemes compared with MT-MAC. We have to perform the deployed test-bad network simulator (MATLAB) platform. The network area is considered in a square 100 × 100, and the field is divided into 10 nodes where start time of each node is 300s running on different sources. We have presented the detail of the parameter in Table 1. We have used constant speed as compared to other different speed mobilities in MAC protocol.

Additionally, each trip of the mobile node is followed by 2s pause time in the RWP model. In the simulation scenario, the average packet delivery ratio and average energy depletion and latency/response time are the main performance parameters.

### 4.3. Average Packet Delivery Ratio

Figures 2-5 show the results of simulation with a different scenario of networks, which have beendeveloped dynamically. The initial experiment shows 6% of whole nodes, which are considered as portable nodes by the velocity among 6 m/s and 21 m/s, and the results have been generated and shown in Figure 2. It is observed from the results that by increasing the mobile/portable node speed the packet delivery ratio reduces while the handover increases.

It has been observed that DT-MAC describes well PDR as compared to MT-MAC, T-MAC, and MS-MAC nearly in all circumstances. It is caused by a mobility strategy that makes it easier for the protocol to manage node movement across virtual clusters. In Figure 2(a), it is also described that entirely protocol achieved higher packet delivery ratio using RWP mobility model where the speed is reached to almost higher than 6%. After each step, the two-pause time random waypoint mobility model is 2 m/s, which provides the protocols higher chance to handover information. In case of random walk mobility model PDR, it will not reduce the pause time and the speed of PDR will definitely increase, which will show more than 11% change in DT-MAC and finally the MT-MAC will get faster.

Figure 3 describes the result of network dynamics on the presentation of the protocols by changing the number of mobile nodes we varied network dynamic level in the network from 0% to 10% whereas 2m fixed speed.

Figure 3also describes the mobile node average PDR which is down up to 10%. DT-MAC illustrates a higher packet delivery ratio from 3 to 7% compared with MT-MAC, MS-MAC, and T-MAC.

The same outline can be detected from the RW mobility model, which is almost 16% PDR, which dropped in T-MAC (Figure 3(b)). The difference between MAC protocol and PDR becomes larger by increasing the number of mobile nodes.

### 4.4. Average Energy Consumption

Figure 4(a) demonstrates how the speed of nodes affects the amount of energy that may be depleted. MT-MAC demonstrates high energy depletion than others, which is due to high energy depletion inside the active zone. It is observed that more nodes are involved by increasing energy depletion. Compared with DT-MAC, MT-MAC is able to reduce the energy depletion from 21% at low speed to more than 66% at high speed. T-MAC demonstrates higher energy usage than DT-MAC due to the lightweight scheme from the transfer, which causes more force power nodes to have additional SYNC and helps for smooth transfer to a new virtual cluster.

Figure 4(b) illustrates the influence of increasing the number of moveable nodes on energy depletion. Here, MT-MAC illustrates more energy depletion among four MAC protocols, whereas DT-MAC enhanced from 26% up to 66% in low dynamic to high network. T-MAC has more energy depletion as compared to DT-MAC, which is due to its enhanced rate of the SYNC method.

### 4.5. Latency/Response Time

The performance of algorithms is evaluated using latency/response time where a better algorithm can be evaluated on better response time/latency as described in Figure 5. The latency of T-MAC is 25 m/secs when the percentage of mobile nodes increased to 10, which results in poor performance. At the same increase in mobile nodes, the latency of MS-MAC is 20 m/secs, which is evaluated as a better response time than T-MAC. Same as the case the DT-MAC results in 7 m/secs, which is evaluated as better than both T-MAC and MS-MAC. MT-MAC results in 5 m/sec response time while increasing the percentage of mobile nodes. Both DT-MAC and MT-MAC algorithms are the same in percentage 3; when increasing to percentage 3, the difference is starting from percentage 10. MT-MAC shows a higher response time as compared to DT-MAC, MS-MAC, and T-MAC.

The simulation results show that a compromise of little latency, roughly 3 percent in using the proposed protocol, eventually improves the MT-MAC's packet delivery by 13–17 percent and the response time by around 15 percent. The more the energy depletion is because more control messages are required for network establishment.

## 5. Conclusion and Future Work

Nowadays, IoT-enabled application has gained the attention in diverse fields including healthcare, underwater sensor network, and body area network [48]. The performance of the proposed algorithm, namely DT-MAC, is compared with well-known algorithms using simulation experiments. Numerous parameters are considered to evaluate the performance of the proposed algorithm such as average packet delivery ratio, average energy depletion, and network response time. The proposed scheme successfully overcomes packet loss and enhanced response, 13%–17% and 15%, respectively, in exchange of compromising 3% energy depletion. It is because of using the idea of “make before break” mechanism of network establishment and maintenance. Moreover, the proposed scheme also planned to reduce gateway nodes that contributed to improving the response time using the idea of minimal dominating set (MDS)-based network formation. Consequently, the proposed method DT-MAC performs better than MT-MAC, T-MAC, and MS-MAC developed methods. The future work is to minimize delay, network maintenance, redundancy, and inconsistency.

## Figures and Tables

**Figure 1:** Display of the formation of DT-MAC from a flat network (G). (a) Flat network. (b) Cluster-based network.

**Figure 2:** (a) Effect of the speed of nodes on the average packet delivery ratio. (b) Effect of the speed of nodes on the packet delivery ratio.

**Figure 3:** (a)Effect of dynamic changes in the PDR. (b) Effect of dynamic changes in the PDR.

**Figure 4:** (a) Effect of node speed on energy depletion (b) Effect of dynamic changes in the energy consumption.

**Figure 5:** Effect of network dynamic ups and downs on the latency/response time.

**Algorithm 1:** Dynamic time scheduling algorithm (DT-MAC).

**Algorithm 2:** Mobility handling phase.

**Table 1:** Simulation parameters.

General topology nodes dispersed equally	Square (150 m × 150 m)
Total nodes	50 nodes
Period	300 s
Data length	up to 512 bytes
Message payload	64 bytes
Duration of data sending	1 packet per second
Mobility model radio with fixed speed	RWP with 2 s pause
Effective data rate	250 kbps
Sleep	1.4 mW
Transmit	62 mW
Receive	62 mW
Tx power output	55.18 mW
Modulation model	PSK

## Data Availability

The data that support the findings of this study are available upon request from the corresponding author.
